RETRACTED

# Noise exposure and its relationship with postinfarction cardiac remodeling: implications for NLRP3 inflammasome activation

**DOI:** 10.1080/21655979.2022.2073126

**Published:** 2022-05-16

**Authors:** Yanzhao Wei, Wei Li, Shuang Yang, Peng Zhong, Yingying Bi, Yanhong Tang

**Affiliations:** a Department of Cardiology, Renmin Hospital of Wuhan University, Wuhan, Hubei, China; b Cardiovascular Research Institute, Wuhan University, Wuhan, Hubei, China; c Hubei Key Laboratory of Cardiology, Wuhan University, Wuhan, Hubei, China; d Department of Cardiology, Wuhan No. 1 Hospital, Wuhan Hospital of Traditional Chinese and Western Medicine, Wuhan, Hubei, China

**Keywords:** Myocardial infarction, noise exposure, purinergic signaling, NLRP3 inflammasome, inflammation

## Abstract

In recent years, high-decibel noise has emerged as a causative risk factor for ischemic heart disease. Massive noise overdose is associated with increased endocrine, neural, and immune stress responses. The NLRP3 (nucleotide-binding oligomerization domain, leucine-rich repeat, and pyrin domain containing 3) inflammasome, the most characterized supramolecular complex and a potent mediator of inflammatory signaling, has been reported to be a marker of increased ischemic heart disease vulnerability. Our study evaluated the association of noise exposure with postinfarction cardiac remodeling and its effect on NLRP3 inflammasome activation. Rats were exposed to a noisy environment (14 days, 24 h/per day, 70 ± 5 dB), and speck formation by the NLRP3 inflammasome scaffold protein ASC (apoptosis-associated speck-like protein) was assessed by confocal immunofluorescence. Echocardiography, pathological analysis, and in vivo electrophysiology were performed. Our results revealed the improved postinfarction cardiac function, mitigated fibrosis, and decreased arrhythmia vulnerability and sympathetic sprouting in low-environment noise groups. Moreover, western blotting of NLRP3, caspase-1, ASC, IL-1β, and IL-18 and confocal microscopy of ASC speck showed that the priming and activation of NLRP3 inflammasome were higher in the NE group than in the NI group. In conclusion, our findings reveal a previously unidentified association between NLRP3 inflammasome activation and noise exposure, underscoring the significance of effective noise prevention in improving postinfarction prognosis.

## Highlights

- Acute surrounding noise insulation after infarction protects against cardiac remodeling compared to a noisy environment.
- ATP-responsive purinergic P2X3 and P2X7 is increased by noise exposure and decreased by noise insulation.
- NLRP3 inflammasome activation is altered subsequent to P2X3/P2X7 alteration.

RETRACTED

## Introduction

Myocardial infarction (MI) is a multifactorial disease with high mortality and morbidity worldwide. Noise pollution, with accelerating urbanization and mechanization, has been reported by the World Health Organization to be the environmental factor with the second most significant environmental risk factor for human health just following air pollution [1,2]. Currently, the guidelines of the ESC and AHA/ASC do not sufficiently address the role of noise as a risk factor for cardiovascular disease, and research on the mechanisms by which noise exposure can lead to cardiovascular disorders is lacking. To date, studies on noise have mainly focused on the ability of long-term exposure to a high sound pressure level to cause direct adverse health effects brought by loud noise such as hearing loss. Furthermore, the non-auditory, indirect noise-related adverse health consequences, firstly described in the 1970s including pain, vision, sleep disturbance, and mental stress, are more profoundly involvedin the noise-induced abnormalities of circulation system. A population-based landmark study in European countries revealed that a noise level over 60 dB is associated with a higher myocardial infarction harard, and it was found by an animal experiment that chronic exposure to a mean sound pressure level about 85 dB leads to 30 mmHg increase in blood pressure in monkeys [3–5]. Previous studies have revealed that noise exposure causes vascular endothelial defects and vasoconstriction, which underlie vulnerability to stress-related heart diseases and hypertension [6–8]. However, few studies have evaluated whether acute exposure in high sound pressure level environment affects postinfarction cardiac remodeling. Elucidating the role of noise exposure in MI progression and underlying its molecular basis are important for clinical practice and hospital management.

Postinfarction inflammatory responses are well defined. Prolonged inflammation has negative consequences, including sympathetic overdrive, alterations in electrophysiological properties, and excessive collagen deposition [9,10]. Sympathetic activation, with stellate ganglia acting as a checkpoint, is pivotal to regulate cardiac inflamamtion [11–13]. ATP (adenosine-5-triphosphate) via P2 purinoreceptors has been validated to induce inflammatory responses under acute sympathetic stress. ATP, upon sympathetic stimulation status, is substantially released into the extracellular space, and enhancing the release of noradrenaline from prejunctional sympathetic nerves [14,15]. Collectively, ATP pathway is involved into the cardiac inflammation after sympathetic overdrive. In addition, ATP is not a major regulator of parasympathetic neural system [16].

RETRACTED

According to the subtypes of NOD-like receptor, the multimeric heterogenous mega-Dalton protein complex namely inflammasome that detects damage-associated molecular patterns, such as ATP, and promote the expression of a plethora of heart failure- and remodeling-associated genes are divided into NLRP1, NLRP3, NLRC4, and AIM2. Among them, the NLRP3 inflammasome is recognized as the most important initiator of aseptic inflammation [17,18]. The active NLRP3 inflammasome reduces the integrity of the cell membrane and the release of proinflammatory mediators, causing persistent, irreversible myocardial damage [19–21]. The NLRP3 inflammasome comprises a sensor protein NLRP3, a scaffold protein ASC, and an effector caspase-1. Upon activation, NLRP3 oligomerizes to recruit ASC. Once ASC recruited, it acts as a ‘catalyst’ to reduce the threshold for caspase-1 activation and the release of IL-1β and IL-18 through the cell membrane pore formed by the gasdermin-D (GSDMD) [22–25]. Remarkably, ASC oligomerization and formation of the scattered, peri-nucleus macromolecule foci, which appear as ASC speck is required for activation of the NLRP3 inflammasome [26]. Detection of ASC specks provide an independent read-out for reduced caspase-1 self-cleavage. Furthermore, canonical activation of the NLRP3 inflammasome occurs via a two-step process. First, in the priming step, necessary proteins are encoded to prepare for NLRP3 inflammasome assembly. In the activating step, the NLRP3 inflammasome is fully assembled. The effector caspase-1 is activated, allowing it to transform IL-1β and IL-18 into their active forms [27]. In our study, we identified NLRP3 inflammasome pathway as the potential target of noise induced cardiac inflammation following acute sympathetic stress. It will be helpful in assessing the impact of noise on the prognosis of acute myocardial infarction patients.

In particular, the potassium efflux through P2X7 receptor induces NLRP3 inflammasome activation [27,28]. Function loss of P2X7 is involved in decreased ischemic heart diseases and hypertension, which are conditions with inflammation [29]. Once activated, P2X7 receptor provides a circular platform for the aggregation of ASC and caspase-1, which cleaves gasdermin-D into fragments to produce a nonselective membrane macropore, through which the components of the NLRP3 inflammasome enter the intracellular space [30]. P2X3 receptor has been shown to cause functional and structural changes of heart innervated sympathetic nerve fibers [31,32]. As a type of neural-specific ATP-gated channels, P2X3 receptor enhances the infiltration of inflammatory cells, amplifies nociceptive sensation and participates in the progression of neuropathy caused by diabetes mellitus and joint arthritis by activating the sympathetic reflex [33,34]. P2X3 receptor is an emerging contributor of inflammation under sympathetic hypersensitive conditions.

RETRACTED

Previous studies have identified the functional and morphological relationships between P2X3 and P2X7 [34–37]. Suppression of one of these receptors leads to a decrease in the expression of the other, and P2X3 receptors and P2X7 receptors show similar expression trends to mediate inflammatory responses [38,39]. Thus, considering the alterations in the expression of P2X3/P2X7 during noise exposure and the tight connection between P2X7 and NLRP3 inflammasome, we speculate that P2X7 and P2X3 somehow work together to modulate NLRP3 inflammasome activation.

The noise-induced sympathetic nervous hyperinnervation, which leads to the release of cortisol and catacholamines, results in the induction of inflammation with increased pro-inflammatory cytokines IL-1β and IL-6. Activated NLRP3 inflammasome responds to sympathetic nervous overdrive by increased IL-1β and IL-18 [40,41]. Herein, we hypothesized that the NLRP3 inflammasome is activated by the P2X3/P2X7 axis in noise exposure environment. Based on this assumption, we assessed the impact of noise exposure on cardiac function and cardiac remodeling. ASC oligomerization, as a specific NLRP3 activation step, was further analyzed. Overall, noise exposure, which induces NLRP3 inflammasome activation, increases cardiac remodeling and boosts inflammation in both stellate ganglia and cardiac tissues.

## Method

### Animal model of noise exposure/insulation and myocardial infarction

All procedures were performed using adult male rats (180 –220 g) according to the Guidelines for the Care and Use of Laboratory Animals published by the US National Institutes of Health (2011, eighth edition, National Research Council) and supervised by Experimental Animal Center of Wuhan University according to the ethical guidelines of the Experimental Animal Center of Wuhan University. All rats were maintained in a specific pathogen-free environment in the Animal Experimental Center of Wuhan University. For the sensitivity of hearing of rats, massive and consistent exposure of 100 dB or more could lead to hear loss, which may cause discrepancy to our study. Herein, in the noise exposure (NE) group, rats were exposed to environmental noise (65 –80 dB) produced by a recording machine in a soundproof box according to the previous study [42]. In the noise insulation (NI) group, rats were arranged with the environmental noise at 25 –35 dB in a soundproof box. The environmental noise was consistent with the daily noise experienced in our cardiovascular ward. Rats in the MI group underwent extra left anterior descending artery ligation after intraperitoneal injection of 2% barbital sodium (40 mg/kg) [43]. ST segment elevation on ECG indicated successful operation. The rats were sacrificed by an overdose of anesthesia on the 14th day after the operation. ECGs were collected for unconscious rats. Stellate ganglia were collected as described in a previous study [44].

RETRACTED

### Cardiac function measurement

The rats were anaesthetized with 2% barbital sodium as previously described and underwent echocardiography under unconscious conditions. Echocardiography was conducted with a Vinno V8 ultrasound machine (Soochow, VinnoTech) and a linear array probe (4 –12 Hz) by a physician working at the imaging department of Wuhan Renmin Hospital. Left ventricular ejection fraction (LVEF), left ventricular fractional shortening (LVFS), left ventricular internal diameter at end-diastole (LVIDd), and left ventricular internal diameter at end-systole (LVIDs) were measure to evaluate postinfarction cardiac function and cardiac structure.

### Masson and sirius red staining

Masson’s trichome staining and Sirius Red staining were used to evaluate the deposition of adipose tissue and collagen in the myocardium. Blood was removed from heart samples, and then the samples were cut transversely into 5 µm slices, fixed in 4% paraformaldehyde solution and embedded in paraffin for staining after deparaffinization and rehydration according to standard procedures [45]. The stained sections were scanned with a NanoZoomer scanner (Hamamatsu Photonics, Japan) and analyzed with NanoZoomer Pathology Digital software NDPview2.0. The Masson’s trichrome- and sirius red-stained areas were analyzed with Fiji ImageJ software. Slices were randomly selected for analysis under a microscope, and six samples from each group were utilized for analysis.

### Caspase-3 activity

The caspase-3 activity was measured by caspase-3 activity assay kit (Beyotime, China, #C1115). According to the for manipulator instruction, the reaction system includes buffer solution, sample, lysis buffer and Ac-DEVD-pNA. After reacting for 120 min, the optical density of 405 –450 nm light absorbance was calculated.

### Immunostaining and confocal analysis of ASC specks

Stellate ganglia and heart tissues were fixed in 4% paraformaldehyde, blocked in 1% fetal bovine serum, and incubated with anti-αSMA antibody (Santa Cruz, USA, #sc-53,142), anti-rabbit GAP43 antibody (Abclonal, China, #A19055), anti-rabbit TH antibody (Abclonal, China, #A0028) anti-rabbit ASC antibody (ImmunoWay, England, YT0365) anti-rabbit αSMA antibody (Abcam, USA, #ab7817) in 0.1% BSA. Then, they were incubated in secondary antibody overnight. After washing and recovery for 1 h, the samples were cut into slices, blocked and observed under a microscope (JAPAN, OLYMPUS). ASC speck was observed by Leica laser scanning confocal microscope (Leica SP-8, Germany).

RETRACTED

### In vivo programmed electrical stimulation (PES)

In vivo PES was conducted after cardiac function measurement under unconscious conditions. First, ECG recording was performed, and assisted respiration by a ventilator was established. Thoracotomy was conducted under aseptic conditions to expose the heart. The ECG baseline parameters QT interval, QTc, PR interval, and QRS wave were analyzed. The duration of arrhythmia was the time from the end of the last burst pace to the first detectable P wave. The data were analyzed with Labchart8 Pro software (AD Instruments).

### RNA extraction and real-time quantitative PCR (qPCR)

Cellular RNA was extracted with TRIzol reagent (Monad, Wuhan) and extracted with trichloromethane according to the manufacturer’s instructions. After processing with dsDNase (Thermo Scientific, USA), the RNA was reverse transcribed into cDNA using a commercial kit from Thermo Scientific Inc. The single-strand cDNA was diluted and amplified for 40 cycles on a PCR machine. mRNA expression was determined by the 2^−ΔΔCT^ method. The primer sequences are listed as follows.

**Table:** 

IL-6	
GCTACCAAACTGGATATAATCAGGA	CCAGGTAGCTATGGTACTCCAGAA
TNF-α	
CACCACCATCAAGGACTCAA	AGGCAACCTGACCACTCTCC
TGF-β	
CCTGAGTGGCTGTCTTTTGACG	AGTGAGCGCTGAATCGAAAGC
IL-10	
GCCAAGCCTTGTCTGAGATGATCC	TTCACATGCGCCTTGATGTCTGG

### Western blotting

Cardiac and dorsal root ganglion tissues were immersed in RIPA lysis buffer after being carefully washed with PBS. The protein concentration in the homogenates was measured with a BCA protein assay kit (Aspen, China, AS1086). The proteins were separated by 10% gel SDS–PAGE until the bromophenol blue ran off the gel and then transferred to a polyvinylidene difluoride membrane. Before incubation with primary antibodies, the membrane was blocked for 1 h at room temperature in 5% fat-free dry milk in PBS. The following primary antibodies were used: anti-rabbit caspase-1 (Abcam, USA, #ab179515), anti-rabbit NLRP3 (Alomono, Israel, #APR016), anti-rabbit ASC (Abcam, USA, #ab260043), anti-rabbit P2X3 (Invitrogen, USA, #PA5-115,707), anti-rabbit P2X7 (Abcam, USA, #ab93354), anti-rabbit P2X4 (Abcam,_USA, #ab168939), anti-rabbit P2X6 (ThermoFisher #PA5-87,659), and anti-rabbit IL-1β (ThermoFisher, USA, #M421B), anti-rabbit NGF (ThermoFisher #PA5-29,425), anti-rabbit GSDMD (Abcam, USA, #ab210070), anti-rabbit collagen I (Abcam, USA, #ab34710), anti-rabbit collagen III (Abcam, USA, #). The membrane was incubated with primary antibody overnight and then with HRP-conjugated goat anti-rabbit IgG (Sungene, China, #LK2001) for 30 min. The membrane was washed, and then the density of the protein bands was quantified using AlphaEaseFC software as described in previous studies [46].

RETRACTED

### Statistical analysis

We calculated the means ± standard errors of the mean (SEMs) to evaluate the data. The normality of the data was assessed by the Shapiro–Wilk test prior to the application of parametric tests. To test the significance of the difference between each group, one‐way analysis of variance (ANOVA) followed by Tukey’s post-hoc test was used. *p* < 0.05 was considered statisticallly significant.

## Results

### Noise insulation preserves cardiac function and suppresses postinfarction myocardial fibrosis

First, in order to explore the effects of noise exposure on cardiac function and cardiac fibrosis, we analyzed echocardiographic images, assessed the pathological sections and the immunofluorescence of fibroblast biomarker αSMA. The noise exposure (NE group) was utilized as the positive control. The rats were divided into four groups: the control and myocardial infarction groups in 35 ± 5 dB environment (CTL+NI, MI+NI), the control and myocardial infarction groups 70 ± 5 dB (CTL+NE, MI+NE). As shown in Figure 1(a-b), LVEF and LVFS were increased and LVIDd and LVIDs were decreased in the MI+NI group (*p* < 0.05) compared to the MI+NE group. Interestingly, the differences in LVEF, LVFS, LVIDd, and LVIDs between the CTL+NE and CTL+NI groups were small (*p* > 0.05). Furthermore, as illustrated by HE staining (Figure 1(c)), Masson’s trichrome staining and Sirius red staining of the left ventricle, collagen deposition was enhanced by MI, but noise insulation prevented the increase in collagen deposition induced by MI. We next examined the myofibroblast activation level using αSMA (Figure 1(d)). The αSMA level was significantly inhibited by noise insulation, particularly in the MI group. Collectively, these results indicate that noise insulation can ameliorate postinfarction cardiac dysfunction and preserve myocardial heterogeneity.

**Figure 1.** Effects of noise on cardiac function and cardiac fibrosis (n = 6 –8 in each group). The data are presented as the mean ±SEM. (a) Representative echocardiographic images. (b) Quantitative analysis of LVEF (%), LVFS (%), LVIDd (mm) and LVIDs (mm). (c) HE staining, Masson’s staining and Sirius red staining were used to evaluate cardiac injury and cardiac fibrosis. (d) Representative images of immunofluorescence staining for the myofibroblast activation biomarker αSMA. *p < 0.05 vs. the MI+NE group.

RETRACTED

### Noise insulation inhibits postinfarction ventricular arrhythmia (VA) vulnerability

In this part, to observe the vulnerability of ventricular arrhythmia, the important end-point event tightly associated with cardiac remodeling, we conducted in vivo programmed electric stimulus and analyzed ECG baseline parameters on ECG recordings. Figure 2(a) shows a representative picture of recorded ECG and PES waves. As shown in Figure 2(b), basic electrocardiographic parameters, including the QT interval, QTc (calculated by Mitchell’s formula), PR, and QRS wave, were similar (*p* > 0.05) between the groups exposed to low- and high-noise environments, indicating that noise did not affect baseline cardiac conduction. However, as shown in Figure 2(c), compared with rats in the MI+NE group, rats in the MI+NI group exhibited reduced VA inducibility (*p* < 0.05) and a shortened VA duration (*p* < 0.05). Moreover, the VA starting time was not obviously different between the NI and NE groups (*p* > 0.05). Overall, the results showed that noise insulation reduces VA vulnerability without affecting baseline cardiac conduction.

**Figure 2.** Effects of noise on VA vulnerability (n = 10 in each group). The data are presented as the mean ±SEM. (a) Representative images of ordinary ECGs and programmed electric bursts for each group captured with Labchart 8.0 software. (b) Quantification of ECG baseline parameters. QT interval, QTc (calculated QT interval based on Mitchell’s formula), PR interval, and QRS interval. (c) VA duration and the onset time to the first VA event after PES. 0s in the figure means there were no VA events after an electric burst. *p < 0.05 vs. the MI+NE group, #*p* < 0.05 vs. the CTL+NE group, **p < 0.01 vs. the MI+NE group, ##*p* < 0.01 vs. the CTL+NE group.

### Noise insulation decreases postinfarction cardiac neural remodeling

Neural remodeling refers to higher level of intramyocardial sympathetic sprouts in border zones of infarcts and altered neurotrophic agents. As we know, the sympathetic hyperinnervation predisposes to ventricular arrhythmia. It was hypothesized that noise exposure increased the susceptibility of ventricular arrhythmia by augmented neural remodeling. To observe the neural remodeling in low and high sound pressure levels, we measured the proteinic levels of sympathetic biomarkers tyrosine hydroxylase (TH) and growth-associated protein 43 (GAP43), and prosurvival nrueal growth factor neural growth factor (NGF) by immunofluorescence and western blotting. Under both sham-operation and MI conditions, a low-noise environment decreased the norepinephrine concentration in heart tissues and the circulatory system (*p* < 0.05), as shown in Figure 3(a). Furthermore, as shown in Figure 3(b), tyrosine hydroxylase and growth-associated protein 43 immunostaining was decreased in rats exposed to a the low-noise environment compared with rats in the CTL group and MI group exposed to a high-noise environment. Moreover, postinfarction augmentation of the protective neurotrophin nerve growth factor NGF in cardiac tissues was relatively canceled (*p* > 0.05) by exposure to sound pressure environment, but not with a statistical significance(Figure 3(c)).

RETRACTED

**Figure 3.** Effects of noise on postinfarction cardiac nervous remodeling (n = 6 –8). The data are presented as the mean ± SEM. (a) Quantification of the local and systemic concentrations of the sympathetic drive biomarker NE (pg/ml). (b) Immunofluorescence staining of the sympathetic nervous system biomarkers TH and GAP43. (c) Western blotting of the anti-remodeling neutrophin NGF and quantification. *p < 0.05 vs. the MI+NE group.

### Noise insulation detains purinergic signaling and ameliorated apoptosis and pyroptosis

Purinergic signaling is a important pathway for cardiac inflammation to promote pyroptosis and apoptosis. Purinergic receptors’ activation derives in inflammation and alteration of cardiac cell viability. In order to verify the impact of noise pressure on programmed cell death, we evaluate the activity of apoptosis-related effector caspase-3 by caspase-3 activity assay and expression level of pyroptosis effector protein gasdermin-D (GSDMD). As shown in Figure 4(a-b), compared with a high-noise environment, noise insulation downregulated GSDMD expression level and cleavage of GSDMD. Besides, the caspase-3 activity kit assay unveiled that the caspase-3 activity of quiet environment group was relatively lower than that of noisy environment group (Figure 4(c)). The TUNEL staining, as depicted in Figure 4(d-f), showed that the TUNEL positive cells under noise insulation group was improved compared with noise exposure group (Figure 4(d-e)).

**Figure 4.** Effects of noise on postinfarction activation of purinergic signaling, cardiac apoptosis and pyroptosis (n = 6 –8). (a) Representative western blotting bands of pyroptosis protein gasdermin D. (b)Quantitative analysis of GSDMD precursor and cleaved form expression level. (c) The illustration of caspase-3 activity assay and its quantitative analysis of caspase-3 activity by optical density. (d) Representative images of TUNEL staining. (e) Representative western blotting bands of P2X3, P2X7, P2X4, P2X6. (f) Quantitative analysis of the percentage of TUNEL positive cells/100 cells. (g) Quantitative analysis of P2X3, P2X7, P2X4, P2X6 expression levels. *p < 0.05 vs. the MI+NE group, **p < 0.01 vs. the MI+NE group.

RETRACTED

To investigate the role of purinergic signaling in noise-related inflammation, we investigated the protein levels of the four major P2X receptors on heart, P2X3, P2X7. P2X4, P2X6 (Figure 4(e-g)). P2X3 and P2X7 expression in cardiac tissues was significantly increased in the NE groups compared with the NI groups (*p* < 0.05). P2X3 and P2X7 expression was decreased in the NI group (*p* < 0.05). However, P2X4 and P2X6 expression was not altered whether under noisy environment. Collectively, it was suggested that noise insulation **r**educed apoptosis and pyroptosis and decreasing P2X3/P2X7 signaling.

### Noise insulation suppresses activation of the NLRP3 inflammasome

The purinergic P2X7 receptor is a key activator of the NLRP3 inflammasome, inducing potassium efflux to trigger the downstream assembly of the NLRP3 inflammasome, and P2X3 has been proven to be synergistic with P2X7. Therefore, after studying P2X3 and P2X7 expression, we investigated the protein levels of NLRP3 inflammasome components and subsequent caspase-1 cleavage and IL-1β maturation in heart tissues and stellate ganglia. As shown in Figure 5(a-b) and quantified in Figure 5(c-d), in cardiac and stellate ganglia tissues, the expression of NLRP3, ASC protein, pro-caspase-1, caspase-1p20 and IL-1β was reduced in low noise group (*p* < 0.05). Notably, according to the results in Figure 5(c-d), the inhibitory effect of noise insulation on the NLRP3 inflammasome was much stronger in MI rats than in CTL rats, and the effects were more significant in heart tissues than in stellate ganglia. Furthermore, ASC specks were observed by confocal immunofluorescence. As presented in Figure 5(e-f), the oligomerization of ASC into speck-like structures was increased upon NLRP3 inflammasome activation. It was clear that the number of stained puncta, i.e. ASC specks, was increased by noise exposure but that ASC speck formation was markedly inhibited by noise insulation.

**Figure 5.** Effects of noise on postinfarction NLRP3 inflammasome activation in heart tissues and cardiac sympathetic ganglia, stellate ganglia (n = 5 –7). (a) Representative western blot bands of NLRP3, ASC, pro-caspase-1, caspase-1p20, and IL-1β in heart tissues. (b) Representative western blot bands of NLRP3, ASC, pro-caspase-1, caspase-1p20, and IL-1β in stellate ganglia. (c) Quantification of the expression levels of NLRP3, ASC, pro-caspase-1, caspase-1p20, and IL-1β in heart tissues. (d) Quantification of the expression levels of NLRP3, ASC, pro-caspase-1, caspase-1p20, and IL-1β in stellate ganglia. (e) Representative images of ASC speck formation; the arrows indicate ASC specks. (f) Quantitative analysis of the percentage of ASC speck positive cell/100 cells. *p < 0.05 vs. the MI+NE group, #*p* < 0.05 vs. the CTL+NE group, **p < 0.01 vs. the MI+NE group, ##*p* < 0.01 vs. the CTL+NE group.

RETRACTED

### Remission of P2X3/7 ameliorated the myocardial injury caused by noise exposure

To further validate the association of purinergic signaling with cardiac inflammation and remodeling consequences resulted from sound pressure, we set myocardial infarction+noise insulation (NI), myocardial infarction+noise exposure (NI), and myocardial infarction+noise exposure+P2X3/7 inhibition (NE+P2X3/7 inhibition) group to evaluate elastic proteins collagen I (col-I), collagen III (col-III), NLRP3 protein, and cytokines IL-6, TNFα, TGFβ, IL-10. It is indicated in Figure 6(a-b) that P2X3/P2X7 inhibition relatively rescued the fibrotic disposition protein col-I (*p* < 0.05) and col-III (*p* > 0.05). Moreover, the anti-inflammatory effect of P2X3/P2X7 inhibition was testified by the decrease of IL-6, TNFα, TGFβ and increase of anti-inflamamtory IL-10 in NE+P2X3/7 inhibition group. The immunohistological staining of NLRP3 also proved that NLRP3 protein could be reduced by antagonized P2X3/P2X7. In this part, it is suggested that different levels of sound pressure very possibly altered postinfarction cardiac injuries by purinergic-involved inflammation.

**Figure 6.** Effects of P2X3/7 inhibition on postinfarction cardiac injuries (n = 5 –7). (a) Representative western blot bands of collagen and collagen III. (b) Quantification of the expression levels of col-I and col-III. (c) Immunohistochemistry staining of NLRP3 protein. (d) qPCR measurement of IL-6, TNFα, TGFβ and IL-10. *p < 0.05 vs. the MI+NE group, #*p* < 0.05 vs. The MI+NI group, **p < 0.01 vs. the MI+NE group, ##*p* < 0.01 vs. the MI+NI group.

## Discussion

According to the WHO, noise pollution is currently the second most important environmental threat to human health, as it increases vulnerability to cardiovascular disorders. A European epidemiological study have revealed that traffic-related noise, the most common type of noise in urban area, is related with the loss of more than 1.6 million healthy life years annually in Western Europe [47]. Our study showed that noise insulation exerts a cardioprotective effect by alleviating NLRP3 inflammasome-induced inflammation in nervous and cardiac tissues. Based on our findings, we describe the possible role of noise in postinfarction cardiac injury on the basis that noise is a cardiovascular risk factor. Our study identifies the specific associations between noise and postinfarction cardiac fibrosis, neural remodeling, ventricular arrhythmia vulnerability and P2X3/P2X7-mediated NLRP3 inflammasome-related inflammation.

RETRACTED

Collagen deposition are major predictors of coronary artery diseases and arrhythmogenesis [48,49]. During this process, ganglia innervated by the heart modulate autonomic nervous system balance and regulate cardiac remodeling. During myocardial ischemia, danger signals that activate sympathetic nerves are secreted, while sympathetic activation maintains high levels of myocardial repair and revascularization. However, excessive, prolonged overactivation of sympathetic nerves cause fibrosis, which induces myocardial stiffness, increased possibility of reentry and delayed repolarization. Ventricular arrhythmia events are the most common complication of MI and one of the major causes of death. The heart is the most ATP-abundant organ, and ATP is an important mediator of P2X receptor activation. Among P2X receptors, P2X7 is the main proinflammatory subtype, and it is expressed on inflammatory cells and intrinsic neurons and mediates potassium efflux through the cellular membrane. In addition, P2X7-mediated potassium efflux not only recruits the P2X3 receptor, the most highly expressed P2X receptor on peripheral nerves, but exacerbates lysosomal fracture, oxidative stress, and mitochondrial defects [50]. K^+^ efflux and the corresponding Ca^2+^ efflux in particular activate NLRP3 inflammasome assembly and accelerate its sebsequent caspase-1-dependent proinflammatory cytokine release [30]. Current literature data validate that P2X7/NLRP3 cascade is one of the most important trigger for cardiac inflammation. Consistent with our hypothesis, in carrageenan-induced NLRP3 activation models, P2X3 and P2X7 expressions and IL-1β and IL-6 levels are simultaneously increased [28,51]. Although it has not been confirmed that P2X3 alone can directly activate the NLRP3 inflammasome, P2X3 activation can promote P2X7-mediated NLRP3 inflammasome activation.

In our experiment, we proved that consistent noise exposure is a risk factor for MI and provided a molecular basis for this phenomenon: signals regulated by the ATP-responding purinergic receptors and P2X7 and P2X3. We found that NLRP3 inflammasome and NLRP3-dependent caspase-1 activation may result from activation of purinergic receptors, further confirming our speculation. Swenja et al. proposed that noise-related sleep fragmentation and circadian alternation induces Nox2-mediated oxidative stress and proinflammatory cytokine expression to impair vascular integrity which is a result from noise induced oxidative and inflammatory responses [52]. However, Laurie et al. confirmed that frequent autonomous arousal and increased cortisol levels due to nocturnal noise are the causative factors of cardiovascular function impairment [53]. Intriguingly, in our experiment, the changes in inflammatory cytokine levels in heart samples in noise exposure and noise insulation environments were much more notable than those in sympathetic ganglia, which indicate the existence of other potential proinflammatory mechanisms apart from the neuroendocrine-cardiovascular axis. Recently, data from the UK Biobank revealed a more complicated association between noise and cardiovascular risk [54]. Glycated hemoglobin levels, blood pressure, body mass index, C-reactive protein levels, and triglyceride levels are relatively higher in people living in an environment of ≥65 Db than in people living in an environment of ≤55 dB, and this effect was not affected by the use of relevant medications. In addition, the gut microbiota-brain-cardiovascular axis has been proven to impair cognitive function, increasing anxiety-like behaviors and decreasing tight junction protein expression. Additionally, noise-induced sleep deprivation is another harzard factor for postinfarction recovery, inducing the oxidative modification of clock genes, which is termed ‘redox control of cellular timekeeping’ [55,56].

RETRACTED

Previous studies, which already highlight the negative effect of postinfarction noise on the patients’ well-being, have yet to well prove the direct associations of noise with the healing process. Besides, earlier studies mostly focused on how long-term chronic exposure to noise (several months or even longer) increases MI vulnerability. In our study, we sought to evaluate the effects of acute noise exposure on the prognosis of MI from the aspect of cardiac neural-inflammation axis. Low sound pressure level exerted cardioprotective effects at least in part by inhibiting the ATP/purinergic receptor/NLRP3 inflammasome pathways in both the heart and heart innervated ganglia. NLRP3 inflammasome assembly and activation steps were suppressed in the noise insulation environment, especially in the context of MI. The expression and oligomerization of the scaffold ASC were decreased in rats in the NI group compared to those in the NE group. Our study first verifies the link between noise sound pressure and the NLRP3 inflammasome activity with P2X3/P2X7 as mediators. The P2X6 and P2X4, which also receive ATP stimuli, were not upregulated, indicating the existence of some inhibitory pathway provoked under noise exposure environment. However, there are some limitations to our work. The holistic mechanism exploration such as RNA sequencing needs to be further validated.

## Conclusion

In conclusion, our data provide evidence that noise insulation alleviates postinfarction cardiac fibrosis and VA, at least in part by decreasing NLRP3-mediated inflammation in ganglia innervated by the heart and local inflammation in the heart. Notably, the decrease in NLRP3 inflammasome activation under noise insulation conditions, which is due to reduced NLRP3 oligomerization and ASC speck formation, may result from downregulation of P2X7/P2X3 receptor expression. Our study reveals the mechanism by which noise exposure acts as a risk factor for postinfarction cardiac stiffness and VA relapse, highlighting that tranquil surroundings are necessary for the heart to recover from ‘big hit events’, such as MI. Thus, noise control measures in the cardiovascular department are warranted.
